# Application and Clinical Value of Machine Learning-Based Cervical Cancer Diagnosis and Prediction Model in Adjuvant Chemotherapy for Cervical Cancer: A Single-Center, Controlled, Non-Arbitrary Size Case-Control Study

**DOI:** 10.1155/2022/2432291

**Published:** 2022-06-15

**Authors:** Yang Wang, Lidan Shen, Jun Jin, Guohua Wang

**Affiliations:** ^1^Department of Physical Examination Center, The Affifiliated Lianyungang Hospital of Xuzhou Medical University, No. 182, Tongguan North Road, Lianyungang 222000, Jiangsu, China; ^2^Department of Obstetrics and Gynecology, Zhangjiagang First People's Hospital, No. 68 Jiyang West Road, Zhangjiagang, Suzhou 215600, Jiangsu, China; ^3^Department of Clinical Laboratory, The Affifiliated Lianyungang Hospital of Xuzhou Medical University, No. 182, Tongguan North Road, Lianyungang 222000, Jiangsu, China; ^4^Department of Obstetrics, The Affifiliated Lianyungang Hospital of Xuzhou Medical University, No. 182, Tongguan North Road, Lianyungang 222000, Jiangsu, China

## Abstract

**Objective:**

A case-control study was conducted to explore the application and clinical value of machine learning-based cervical cancer (CC) diagnosis and prediction model in adjuvant chemotherapy of CC.

**Methods:**

From August 2019 to August 2021, 46 patients with stage IA CC (study group) and 55 patients with high-grade squamous intraepithelial lesions (HSIL) (control group) were retrospectively analyzed. All patients completed routine MRI examinations, the ADC values of diseased CC and normal cervix and cervical tissues in different stages were compared, and the changes of ADC values in CC tissues before and after chemotherapy were analyzed. The training set (IA = 37, HSIL = 44) and test set (IA = 9, HSIL = 11) are set in a ratio of 4 : 1. The preoperative MRI images were collected and uploaded to the radiomics cloud platform after preprocessing, and the cervix was manually delineated layer by layer on OSag-T2WI, OAx-T1WI, and OAx-T2FS, respectively, to obtain a three-dimensional volume of interest (VOI) of the cervix to extract omics features. Variance Threshold analysis, univariate feature selection (SelectKBest), and least absolute shrinkage and selection operator (LASSO) are adopted to reduce the dimension of data and enroll features. The arbitrary forest model was adopted for machine learning, the ROC curve was drawn, and the diagnostic performance of different sequence omics models was analyzed.

**Results:**

Compared with ADC of stage A CC and HSIL, the ADC value of CC was remarkably lower than that of normal CC (*P* < 0.05). The ROC curve analysis of ADC value to differentiate CC and normal cervix indicated that the AUC was 0.838 and the 95% confidence interval was 0.721–0.955. According to the maximum Youden index of 0.848, the optimal critical value of ADC was 1.267 × 10^−3^ mm^2^/s and the sensitivity and specificity were 92.21% and 9.48%, respectively. All results are indicated in Table 2. After CC treatment, 12 patients were effective (CR + PR) and 4 patients were ineffective (PD + SD). When the *b* value was 1000 s/mm^2^, the ADC value of the effective patients after the second chemotherapy was significantly higher than that of the first chemotherapy and before treatment (*P* < 0.05). There was no significant difference between the ADC value after the first chemotherapy and before treatment, compared with before treatment (*P* > 0.05). There was no significant difference in ADC value between the ineffective patients before treatment and after the first and second chemotherapy (*P* > 0.05). A total of 8 omics features were extracted based on OSag-T2WI, all of which were wavelet features, including 7 texture features and 1 first-order feature. A total of 10 omics features were extracted based on OAx-T1WI, including 6 wavelet first-order features, 2 gradient first-order features, and 2 wavelet texture features. Based on OAx-T2FS, 6 omics features were extracted, including 3 wavelet texture features, 2 original shape features, and 1 logarithmic first-order feature. Based on OSag-T2WI&OAx-T2FS, 9 histological features were extracted, 4 from OSag-T2WI and 5 from OAx-T2FS. The diagnostic performance of the four arbitrary forest models is indicated in Table 1, and the ROC curve is indicated in Figure 6. The diagnostic performance of the omics model based on OSag-T2WI&OAx-T2FS was the best in both the training set and the test set. The AUC of the training set was 0.991 (95% CI (0.94, 1.00)), and the accuracy rate was 0.925. The AUC of the test set was 0.894 (95% CI (0.75, 1.00)), and the accuracy rate was 0.835. On the other hand, the diagnostic efficiency of the group model based on OAx-T1WI was the worst in both the training set and the test set. The AUC of the training set was 0.713 (95% CI (0.52, 0.92)), and the accuracy rate was 0.71. The AUC of test set is 0.513 (95% CI (0.24, 0.77)), and the accuracy rate was 0.56, which has no practical clinical significance.

**Conclusion:**

A CC diagnosis and prediction model based on machine learning can better distinguish stage IA CC from HSIL in the absence of clear lesions, which is of great significance for reducing invasive examination before surgery, guiding surgical procedures and adjuvant chemotherapy for CC.

## 1. Introduction

With the continuous improvement of material living standards in modern society, the living environment and lifestyle of human beings have also undergone corresponding changes and the accompanying cancer problem has become the most serious problem threatening human health [1]. According to estimates from the “Global Cancer Incidence and Mortality 2018” (GLOBOCAN2018) data compiled by the International Agency for Research on Cancer, there were approximately 18.1 million new cancer cases and 9.6 million cancer deaths in 2018. According to the Surveillance, Epidemiology, and End Results Program (SEER) project, in 2019, about 1.8 million people in the United States was diagnosed with cancer, and meanwhile, 606,880 people passed away from cancer [2]. An estimated number of 268,600 women and 2,670 men were diagnosed with breast cancer, the most common cancer. Compared with other cancers, CC ranks at the forefront among the cancers that affect women's health, especially in areas with backward economic development. Due to the lack of medical resources and the backward medical level, most women rarely have the opportunity to be vaccinated with HPV. vaccines and surgeries or related cancer drugs are rarely performed or administered after the disease, so the morbidity and mortality of the disease are higher than in developed regions. In recent years, the incidence and mortality of CC have been on the rise, especially among middle-aged and elderly women. Therefore, it is necessary to standardize the diagnosis and treatment of CC and enhance the prognosis of patients with CC.

Over the past few decades, researchers have taken different approaches to diagnosing the type of cancer before it becomes symptomatic [3]. Traditional cancer diagnosis methods usually use cell morphology, histopathology, and other methods, but traditional cancer diagnosis methods usually cannot meet the requirements of early diagnosis and early treatment required by clinical practice. With the gradual emergence of new technologies in the field of machine learning, machine learning has been applied in different fields and in different scopes, such as advertising, insurance, finance, social media, and fraud detection [4]. At the same time, a large number of cancer data have been collected and provided to the machine learning research community. Compared with traditional cancer diagnosis methods, machine learning does not use explicit instructions but relies on pattern recognition and reasoning to discover and identify specific patterns from complex datasets, which can effectively predict cancer. However, accurate prediction of cancer outcomes remains one of the most interesting and challenging tasks currently in the field of machine learning. Cancer diagnosis prediction includes three prediction tasks: (1) cancer susceptibility prediction; (2) cancer survival prediction; (3) cancer recurrence prediction [5]. In the first two cases, the first is to try to discover the likelihood that the disease will evolve into a cancer and the second is to predict a survival outcome, such as how long a patient will survive. In the last case, it is to predict the likelihood of developing a cancer after a complete or partial remission of the disease.

When experts formulate a diagnosis and treatment plan for CC patients, they usually predict based on their past diagnosis and treatment experience or search for medical records similar to the current patient in the computer. At each stage of the treatment of CC patients, experts need to consider many factors, such as the stage of CC, whether to preserve fertility, whether there are high-risk factors for recurrence after surgery (parauterine invasion, deep stromal invasion, or lymph node invasion), and lymph node metastasis status [6, 7]. The effect of disease diagnosis and treatment is affected by the medical level of doctors. The process of formulating a diagnosis and treatment plan is based on past experience and the current situation of patients and is subject to a certain degree. Especially for areas with backward medical standards, it affects patients to a certain extent.

HSIL is considered a precancerous lesion of CC, and stage IA CC is an early stage that can only be diagnosed by microscopy [1, 8]. The surgical methods of the two are quite different. HSIL is mainly based on cervical conization. In principle, total hysterectomy is required for stage IA CC (extrafascial hysterectomy for stage IA1, modified extensive hysterectomy, and pelvic hysterectomy for stage IA2) [9, 10]. Therefore, the accurate identification of the stage of the disease before operation is of great significance to the choice of operation mode and scope. However, the scope of lesions in stage IA CC and HSIL is often limited on MRI images, and it is often difficult to identify them with naked eyes, which leads to the limited value of conventional MRI images in the recognition of both. In recent years, with the rise of imaging science research, the information reflected by images is no longer limited to morphological changes and the data potential behind it has been gradually excavated and utilized. As a recent innovation in medical image analysis, imaging technology can extract quantitative features from medical images with high throughput, thus transforming visual images into computable data [11–13]. There has been a lot of practice to combine the imaging data with machine learning to analyze the cervical lesions which are difficult to be recognized by the naked eye. In this study, the histological features of cervix were extracted from magnetic resonance images and a machine learning model was established with arbitrary forest algorithm (RF) to explore the role of imaging techniques in distinguishing stage IA CC from HSIL. The application and clinical value of the machine learning-based CC diagnosis and prediction model in adjuvant chemotherapy of CC were analyzed.

## 2. Patients and Methods

### 2.1. General Information

Forty-six patients with stage IA CC treated in our hospital from August 2019 to August 2021 were enrolled. All patients were confirmed as having advanced primary CC by operation and pathology or cervical biopsy, and no radiotherapy, chemotherapy, or operation was performed before imaging examination. The age ranged from 28 to 69 years, with an average age of (46.02 ± 7.42) years; 28 cases of squamous cell carcinoma and 18 cases of adenocarcinoma were treated with NACT after the diagnostic examination, and MRI examination was performed again after the first and second chemotherapy, respectively. Another 55 patients with HSIL were enrolled as the normal control group, aged 29–65 years, with an average age of (45.31 ± 7.42) years. There was no significant difference in general data such as age and body weight (*P* > 0.05), which was comparable. This study was permitted by the medical ethics committee of our hospital, and the subjects were exempted from informed consent.

Selection criteria were as follows: (1) patients with HSIL or stage IA CC confirmed by pathology during or after operation; (2) patients who did not receive any treatment before operation; (3) MRI examination was performed in our hospital before operation, the image quality was good, and there was no obvious artifact.

Exclusion criteria were as follows: (1) there is a cervical capsule; (2) there is cervical leiomyoma or low uterine leiomyoma involving cervical myometrium; (3) there are congenital malformations in the upper part of the cervix or vagina.

### 2.2. Treatment Methods

#### 2.2.1. The Method of Treatment and the Judgment of Curative Effect

Total intravenous neoadjuvant chemotherapy (NACT): cisplatin 50 mg/m ∼ 2 + Isu 75 mg/m^2^ was given for one day, hydration treatment was performed before and after chemotherapy, and the second course of treatment was performed after 2 weeks. After two courses of treatment, the curative effect was judged according to the latest international criteria for evaluating the curative effect of solid tumor: (1) complete response (CR) tumor disappeared completely; (2) the maximum diameter of partial response (PR) tumor (measured on conventional MRI T2WI) decreased by at least 30%; (3) the maximum diameter of disease progression (PD) tumor increased by 20% or more; (4) stable disease (SD) was between PR and PD. According to the clinical efficacy after treatment, patients were assigned to effective group (CR + PR) and ineffective group (PD + SD).

#### 2.2.2. Image Acquisition

Images were acquired by scanning with a 3.0T MR device (GEDiscoverySilent750 W). The scanning parameters of the equipment are as follows: OSag-T2WI (propeller sequence, TR4390 ms, TE90 ms), slice thickness 4 mm, slice interval 1 mm, field of view 260 mm × 260 mm, matrix 320 × 320; OAx-T1WI (FSE sequence, TR810 ms, TE9 ms) and OAx-T2FS (propeller sequence, TR4530 ms, TE80 ms), layer thickness 5 mm, layer spacing 1 mm, field of view 260 mm × 260 mm, matrix 384 × 384. Images are copied in DICOM format (patient information removed).

#### 2.2.3. Image Preprocessing and Segmentation

Copied images were preprocessed using the Simple ITK package in Python (version 3.8). The N4 bias field correction is adopted to eliminate grayscale differences caused by local magnetic field inhomogeneities; the resampling uses a linear interpolation algorithm and a nearest neighbor interpolation algorithm to achieve uniform and isotropic voxel size. The preprocessed images were uploaded to the radiomics cloud platform (Huiying Medical Technology Co., Ltd., Beijing). The flow chart of radiomics processing is indicated in Figure 1. The entire cervical region is employed as the ROI. The axial plane is delineated layer by layer along the cervical border and finally fused into a VOI. In sagittal delineation, there is a delineation from the second layer that appears on one side of the cervix to the previous layer where the contralateral cervix disappears and a delineation along the 2 mm area outside the border at the external cervical part; in axial delineation, the layer that appears from the upper cervix is delineated and the second layer is drawn to the layer after the cervix disappears.

#### 2.2.4. Feature Extraction

1409 omics features including first-order features, shape features, texture features, and high-order features in VOI are extracted. Texture features include gray-level dependence matrix (GLDM), gray-level co-occurrence matrix (GLCM), gray-level size zone matrix (GLSZM), gray-level run length matrix (GLRLM), and neighboring gray tone difference matrix (NGTDM). Higher-order features are logarithm, exponential, gradient, square, square root, and wavelet transform for first-order features, shape features, and texture features, among which wavelet includes LLL, LLH, LHL, HLL, LHH, HLH, and HHL.

#### 2.2.5. Feature Selection

The data were successively subjected to dimension reduction and selection using Variance Threshold method, single variable feature selection method (SelectKBest), and leaf absolute shrinkage and selection operator (LASSO) regression. Among them, the Variance Threshold enrolls the feature with the threshold >0.80, the SelectKBest enrolls the feature with *P* < 0.05, and the LASSO regression enrolls the most valuable feature based on the coefficient of the optimal alpha.

#### 2.2.6. Machine Learning

Using the RF model, the eigenvalues of each sequence filtered by LASSO regression were included in the calculation. The training set (IA = 34, HSIL = 41) and the test set (IA = 9, HSI = 10) were set according to the ratio of 4 : 1. Based on the eigenvalues extracted by OSag-T2WI, OAx-T1WI, OAx-T2FS, and OSag-T2WI&OAx-T2FS, four RF models were established, and ROC curves of the test set were drawn to test the diagnostic efficiency of the models. The specificity and sensitivity at the optimal cutoff point (maximum Youden index) were chosen.

#### 2.2.7. Statistical Analysis

All data were analyzed with SPSS17.0 statistical software, measurement data were expressed in the form of *x* ± *s*, measurement data between groups were compared by the *t* test, and count data were calibrated by the *χ*^2^ test. The area under the receiver operating characteristic (ROC) curve (AUC) was adopted to analyze the value of ADC values in diagnosing CC. *P* < 0.05 was considered statistically significant.

## 3. Results

### 3.1. Comparison of ADC of Stage IA CC and HSIL

First, we compared ADC of stage IA CC and HSIL. The ADC value of CC was statistically lower than that of normal CC (*P* < 0.05). All results are indicated in Table 1.

### 3.2. ROC Curve Analysis of ADC Value in the Diagnosis of CC

We analyzed the diagnostic value of using ROC curve to distinguish CC from the normal cervix. The results indicated that AUC was 0.838, 95% confidence interval was 0.721∼0.955, the maximum value of Youden index was 0.848, the best critical value of ADC was 1.267 × 10^−3^ mm^2^/s, and the sensitivity and specificity were 92.21% and 9.48%, respectively. All the results are indicated in Table 2.

### 3.3. Comparison of ADC Values of Patients in Different Treatment Groups at Different Time Points before and after Treatment

After CC treatment, 12 patients showed effect (CR + PR) and 4 patients did not show effect (PD + SD). When the *b* value was 1000 s/mm^2^, the ADC value of the effective patients after the second chemotherapy was statistically higher than of the first chemotherapy and before treatment *P* < 0.05(*P* < 0.05); the ADC value after the first chemotherapy was not statistically different from that before treatment (*P* > 0.05). There was no significant difference between the ADC values of ineffective patients before treatment and after the first and second chemotherapy (*P* > 0.05). The specific results are indicated in Table 2.

### 3.4. Model Building

We built a diagnosis and prediction model of CC based on machine learning. The specific results of imaging feature screening are as follows: 8 ensemble features are extracted based on OSag-T2WI, all of which are wavelet features, including seven texture features and one first-order feature. A total of 10 combinatorial features are extracted based on OAx-T1WI, including 6 wavelet first-order features, 2 gradient first-order features, and 2 wavelet texture features, and 6 combinatorial features are extracted based on OAx-T2FS, including 3 wavelet texture features, 2 original shape features, and 1 logarithmic first-order feature. Nine histological features were extracted based on OSag-T2WI&OAx-T2FS, four from OSag-T2WI and five from OAx-T2FS. Specific results are indicated in Figures 2–5.

### 3.5. Comparison of Diagnostic Efficiency of Stochastic Forest Models with Different Sequences

We compared the diagnostic efficiency of different sequence arbitrary forest models. The diagnostic efficiency of the four arbitrary forest models is indicated in Table 1, and the OSag-T2WI&OAx-T2FS-based ROC curve is indicated in Figure 6. The diagnostic efficiency of the combinatorial model based on ROC is the best in both training and test sets. The AUC of the training set was 0.991, with 95% CI of (0.94, 1.00), and the accuracy rate was 0.925. The AUC of the test set was 0.894, with 95% CI of (0.75, 1.00), and the accuracy rate was 0.835. The diagnostic efficiency of the omics model based on OAx-T1WI was worst in both the training set and the test set. The AUC of the training set was 0.713, with 95% CI of (0.52, 0.92), and the accuracy rate was 0.71. The AUC of the test set was 0.513, with 95% CI of (0.24, 0.77), and the accuracy rate was 0.56, which has no practical clinical significance. All the results are indicated in Table 3 and Figure 6.

## 4. Discussion

In the past decade, a variety of different techniques and algorithms have been widely adopted for disease prediction [12]. Most of these studies use machine learning methods to model and identify informative factors, which are then employed in classification schemes. The success of disease diagnosis depends on the quality of medical diagnosis. Improving the quality of medical diagnosis is the ultimate goal of machine learning and intelligent medicine. Major machine learning techniques, including neural networks and decision trees, have been adopted in cancer detection. Many machine learning techniques have been applied to the medical diagnosis of cancer, such as CC, breast cancer, prostate cancer, and lung cancer. According to Court et al.'s findings on machine learning and cancer retrieved from PubMed, more than 7510 related articles have been published to date [13]. The vast majority of these articles uses one or more machine learning algorithms and integrates data from different sources for tumor detection and cancer type prediction.

Over the past decade, the application of supervised learning techniques in cancer prediction has indicated an increasing trend and classification algorithms are widely adopted in various problems posed in cancer research. Shi introduced the application of machine learning in medical images, mainly including the use of machine learning techniques to solve practical problems in “image recognition of lung cancer pathological cells” and “prostate CT image segmentation” [14]. Yu proposed a method combining transfer learning with convolutional neural network, which has a good effect in cancer image recognition [15]. Lv proposed a support vector machine-based pancreatic cancer detection method and found 12 characteristic genes closely related to pancreatic cancer [16]. Ning et al. applied semisupervised learning of graph convolutional networks to predict whether a patient had cancer [17]. Wu and Zhou proposed two improved support vector machine methods, SVM-PCA and SVM-RFE, for the diagnosis of CC [18]. They used a dataset of 858 cases, each containing 32 predictor variables and 4 target variables. Due to the imbalance of the dataset, oversampling was adopted during preprocessing, after which 668 records were enrolled for analysis. The results indicate that SVM-PCA outperforms SVM-RFE. When using SVM-RFE for prediction, the authors also listed the top 10 relevant characteristics of the 4 target variables, such as years of hormonal contraceptive use and smoking. In the past, typical information used by physicians included histological, clinical, and population-based data to make sound judgments about cancer prediction. Diet, weight, family history, age, high-risk habits, and exposure to environmental carcinogens play a key role in predicting cancer development.

Ayer et al. used a neural network approach to risk assessment of the likelihood of developing breast cancer [19]. The data adopted by the authors included mammograms and demographic characteristics. In the study, the neural network was adopted as a predictive model to find radiographs of patients with malignant breast cancer in a mixture of radiographs and to classify patients with benign breast cancer from those with malignant breast cancer. They build models with a large number of hidden layers, which are more accurate than networks with a small number of hidden layers. Data collected for the study included 48,774 mammograms, as well as demographic risk factors and tumor characteristics. All mammograms were reviewed by a radiologist, and labeling information was obtained. The authors then use this dataset to train a neural network model and evaluate its performance through ten-fold cross-validation. Furthermore, to prevent overfitting, the authors use the Early Stopping method. In general, this method reduces errors during training and stops when overfitting occurs. After training and testing with ten-fold cross-validation, the model has a calculated AUC of 0.965. The authors believe that if trained on a large amount of data, their model will be able to accurately assess breast cancer risk.

Early identification of cervical lesions is of great significance, not only to save the patient's life but also to maximize the preservation of the patient's reproductive function [20]. At present, for stage IA CC and HSIL, the “three-step” procedure of cervical cytology and high-risk human papillomavirus (HPV) DNA detection, colposcopy, and cervical biopsy is still used. There is not yet a noninvasive test that can tell the two apart. For cervical lesions beyond stage IA, traditional MRI can assess the extent of invasion, lymph node involvement, and distant metastasis, thereby helping staging [21]. However, for stage IA CC and HSIL, the changes reflected in the images are often at the millimeter level or even sub-millimeter level, and there is a large error in the recognition of the human eye. After the combination of radiomics and artificial intelligence, small differences that cannot be recognized by the naked eye can be found, which is noninvasive and convenient, and it has good patient compliance, which has practical research significance.

Stage IA CC is a lesion with an invasion depth of less than 5 mm, the lesions of HSIL are more limited, and it is difficult to observe the existence of both on MRI images with the naked eye [22]. Therefore, the cervix was delineated as an ROI. In order to prevent the extraction of too many nonstrong features from interfering with modeling, when delineating in the sagittal plane, the delineation layer removes the layers where the cervix begins to appear on the left and right sides, because these two layers often contain more parametrial tissue, which will cause the volume effect and, in the same way, removes the layer of the upper cervix and uterus junction when delineating in the axial position. Meanwhile, given that the most common site of CC is the mucosal transition zone of the external cervical part, in order to maximize the inclusion of the lesions in the ROI, when delineating the sagittal view, the external cervical partwill be delineated to 2 mm outside the boundary [23]. The observed area is delineated along the cervical border, and the axially observed area needs to be drawn to the level after the cervix disappears. This segmentation can not only incorporate the lesion into the ROI as much as possible when it is difficult for the naked eye to identify where it is but also reduce the computational burden caused by the large delineated area. The final generated VOI, as a three-dimensional image, can more comprehensively reflect the heterogeneity of the tissue and enhance the diagnostic efficiency of the model.

In this study, the AUC values of the training set and test set of the arbitrary forest model established based on OAx-T1WI eigenvalues were not ideal. The AUC of the test set was only 0.513, which was equivalent to arbitrary guessing and had no discriminant value. The authors speculated that it was imaging. The sequence and eigenvalue types cause the model to underfit. Roy et al. collected three groups of T1WI and T2WI images of breast cancer patients with different resolutions, and based on this, they generated multiple groups of MRI images with different signal-to-noise ratios [23]. Values are more susceptible to changes in signal-to-noise ratio than T2WI. In this experiment, 80% of the 10 omics feature values extracted based on OAx-T1WI were first-order features. First-order features are simple statistical features that convert VOI into a single histogram to describe the distribution of voxel intensities and derive from them parameters such as Energy, Entropy, Range, and Skew Eigenvalues such as Skewness. These feature values are simple and easy to extract, but not as reliable as texture features. This was also confirmed by the experiments of Mu et al. [24]. In their experiments, there were differences in first-order features such as Entropy and standard uptake value kurtosis (SUVpeak) in early and advanced CC, based on their established support. The vector machine (SVM) model AUC values are all lower than texture features, and the AUC (0.625) of SUVpeak is the lowest among all feature values. In summary, the authors believe that the first-order eigenvalues extracted based on the OAx-T1WI sequence may not be strong features, which will lead to underfitting of the model, so the OAx-T1WI is not adopted to construct a joint analysis model.

Texture features are extracted from different descriptive matrices, which can reflect the correlation between different voxels in a given image and capture the spatial relationship between adjacent voxels, so it has important value in studying tissue heterogeneity. In this experiment, the texture eigenvalues mainly come from the following three groups: GLDM describes the number of voxels with similar gray values within a certain distance centered on a voxel and is a matrix representing the surrounding correlation; GLRLM defines the length of continuous voxels with the same gray value in different directions, reflecting the thickness and uniformity of the image texture; GLSZM quantifies the characteristics of the gray area in the image, which can measure the voxels in the image [25, 26]. The uniformity of gray distribution is a group of texture features that are frequently used in medical imaging research. Before that, no one has used the omics model to predict the stage IA CC and HSIL. Guo et al. assigned CC into early stage (stage IB and stage II) and advanced stage (stage III and stage IV) according to FIGO staging [27]. In the two groups, the GLRLM-based SVM model has the highest AUC (0.88) and the GLSZM (AUC = 0.764) is slightly second. The most ideal model in this experiment is GLRLM (AUC = 0.89). The texture features are mainly from GLSZM. So far, it has been empirically verified that the degree of gray level quantization has an important impact on texture classification performance. Therefore, GLSZM is more effective in characterizing texture consistency and aperiodic or speckle texture than GLDM and GLRLM and has better performance on the texture of nuclei and PET images. In addition to being used to predict staging, GLRLM has also been indicated to predict postoperative recurrence of CC. Interestingly, some studies have found that GLRLM is less reproducible and unreliable in the omics features of CC. Roy et al.'s experiments also seem to confirm this point. They think that GLRLM is the most sensitive texture feature to the change of signal-to-noise ratio and there is no unified conclusion.

The eigenvalues screened in this study also include GLDM, but it has not been found to be related to CC staging in the previous literature [28]. The authors speculate that it is related to the way ROI is delineated. The invasiveness of HSIL is different from that of stage IA CC. The former is confined to the epithelial layer and has not yet penetrated the basement membrane, while the latter penetrates through the basement membrane and infiltrates the interstitial layer. There is a fundamental difference in the transition zone at the edge of the lesion, and GLDM is exactly the A matrix representing the correlation between the center voxel and surrounding voxels. Guo et al. found that GLDM was an important feature for predicting myometrial invasion in endometrial cancer [27]. Yu et al. also found that GLDM was highly correlated with the expression level of Ki-67 in breast cancer tissues and Ki-67 was closely related to the expression of tumor cells [28]. Growth infiltration and lymph node metastasis are closely related. Previous experiments tended to focus more on the lesion itself, while ignoring the relationship between it and normal tissue. The ROI in this experiment has a wide range and can fully reflect the texture features around the lesion.

The ROC curve was adopted to analyze the diagnostic performance of ADC value for CC. According to the maximum Youden index, the ADC value of 1.267 × 10^−3^ mm^2^/s was enrolled as the best critical value, which has high diagnostic performance. In addition, this study found that the difference in ADC value of CC in different stages was significant, indicating that in addition to distinguishing CC from normal cervix, DWI can also be employed to indicate disease staging and provide a reference for evaluating the malignancy of CC. Due to the small number of included cases, this study did not study the threshold value of ADC value for diagnosing different stages of CC and further studies are needed to collect further cases.

In this study, it was found that the ADC value of the effective group increased slightly after the first chemotherapy and the ADC value increased significantly after the second chemotherapy; while the ADC value of the patients in the ineffective group changed after the first and second chemotherapy. It is not obvious suggesting that the application of DWI to detect the changes of ADC value in CC patients before and after NACT treatment can dynamically monitor the chemotherapy efficacy, which has potential clinical application value for the prediction of CC chemotherapy efficacy.

Conclusively, the arbitrary forest model based on MRI imaging can better distinguish stage I A CC from HSIL without obvious lesions, which has certain clinical significance in reducing preoperative invasive examination and guiding CC adjuvant chemotherapy.

## Figures and Tables

**Figure 1:** ROC curve analysis of ADC value in differentiating CC from the normal cervix.

**Figure 2:** Histological characteristics based on OSag-T2WI.

**Figure 3:** Histological features based on OAx-T1WI.

**Figure 4:** Omics characteristics based on OAx-T2FS.

**Figure 5:** Histological features based on OSag-T2WI&OAx-T2FS.

**Figure 6:** ROC curve of the arbitrary forest test set. Note: A: OSag-T2WI; B: OAx-T1WI; C: OAx-T2FS; D: OSag-T2WI & OAx-T2FS.

**Table 1:** Comparison of ADC of stage IA CC and HSIL ($\bar{x}\pm s$).

Group	*N*	Pathological results	*t*	*P*

R group	46	0.91 ± 0.17	17.220	<0.01
C group	55	1.49 ± 0.16		

**Table 2:** Comparison of ADC values at different time points before and after treatment in patients with different curative effects ($\bar{x}\pm s$, ×10^3^ mm^2^/s).

Group	*N*	Before treatment	One week after operation	2 weeks after operation

Effective	12	0.91 ± 0.14	1.02 ± 0.16	1.24 ± 0.38^ab^
Invalid	4	0.91 ± 0.16	1.03 ± 0.12	1.02 ± 0.27
*t*		0.000	0.114	1.061
*P*		＞0.05	＞0.05	<0.01

*Note.* ^a^Compared with before treatment, *P* < 0.05; ^b^compared with the first chemotherapy, *P* < 0.05.

**Table 3:** Diagnostic efficiency of arbitrary forest models with different sequences.

Model		Test set				Training set			
		AUC	95% CI	Sensitivity degree	Specificity degree	AUC	95% CI	Sensitivity degree	Specificity degree

OSag-T2WI									
	HSIL	0.851	(0.68, 1.00)	1.00	0.58	0.971	(0.92, 100)	0.92	0.95
	IA	0.851	(0.68, 1.00)	0.58	1.00	0.971	(0.92, 100)	0.95	0.92

OAx-T1WI									
	HSIL	0.513	(0.24, 0.77)	0.57	0.57	0.713	(0.52, 0.92)	0.76	0.68
	IA	0.513	(0.24, 0.77)	0.57	0.57	0.713	(0.52, 0.92)	0.68	0.76

OAx-T2FS									
	HSIL	0.832	(0.61, 1.00)	0.79	0.90	0.943	(0.88, 1.00)	0.88	0.89
	IA	0.832	(0.61, 1.00)	0.90	0.79	0.943	(0.88, 1.00)	0.89	0.88

OSag-T2WI&OAx-T2FS									
	HSIL	0.894	(0.75, 1.00)	0.79	0.90	0.991	(0.94, 1.00)	0.94	0.93
	IA	0.894	(0.75, 1.00)	0.90	0.79	0.991	(0.94, 1.00)	0.93	0.94

*Note.* HSIL: high-grade squamous intraepithelial lesion; IA: CC (stage IA); OSag: sagittal view; OAx: axial view; FS: fat-suppressed sequence.

## Data Availability

No data were used to support this study.
